This article has been retracted.

# Circulating plant miRNAs can regulate human gene expression *in vitro*

**DOI:** 10.1038/srep32773

**Published:** 2016-09-08

**Authors:** Chiara Pastrello, Mike Tsay, Rosanne McQuaid, Mark Abovsky, Elisa Pasini, Elize Shirdel, Marc Angeli, Tomas Tokar, Joseph Jamnik, Max Kotlyar, Andrea Jurisicova, Joanne Kotsopoulos, Ahmed El-Sohemy, Igor Jurisica

**Affiliations:** 1 IBM Life Sciences Discovery Centre, Princess Margaret Cancer Centre, University Health Network, Toronto, Ontario, Canada; 2 Lunenfeld Tanenbaum Research Institute, Toronto, Ontario, Canada; 3 Department of Obstetrics and Gynecology, Physiology, University of Toronto, Toronto, Ontario, Canada; 4 CRO Aviano National Cancer Institute, Cancer Bio-Immunotherapy Unit, Aviano, PN, Italy; 5 Department of Nutritional Sciences, Faculty of Medicine, University of Toronto, Toronto, Ontario, Canada; 6 Women’s College Research Institute, Women’s College Hospital, Toronto, Ontario, Canada; 7 Dalla Lana School of Public Health, University of Toronto, Toronto, Ontario, Canada; 8 Departments of Medical Biophysics and Computer Science, University of Toronto, Toronto, Ontario, Canada; 9 Institute of Neuroimmunology, Slovak Academy of Sciences, Bratislava, Slovak Republic

## Abstract

While *Brassica oleracea* vegetables have been linked to cancer prevention, the exact mechanism remains unknown. Regulation of gene expression by cross-species microRNAs has been previously reported; however, its link to cancer suppression remains unexplored. In this study we address both issues. We confirm plant microRNAs in human blood in a large nutrigenomics study cohort and in a randomized dose-controlled trial, finding a significant positive correlation between the daily amount of broccoli consumed and the amount of microRNA in the blood. We also demonstrate that Brassica microRNAs regulate expression of human genes and proteins *in vitro*, and that microRNAs cooperate with other Brassica-specific compounds in a possible cancer-preventive mechanism. Combined, we provide strong evidence and a possible multimodal mechanism for broccoli in cancer prevention.

Vegetables and fruits are important components of a healthy diet with a broadly recognized beneficial effect on human well-being. Their intake has been associated with prevention of many diseases including coronary heart disease, rheumatoid arthritis, chronic obstructive pulmonary disease, asthma, osteoporosis, dementia, and most notably, cancer^1^. Numerous epidemiological studies specifically highlighted an important disease prevention role of cruciferous vegetables (e.g., Brassicaceae)^2^. Findings from several meta-analyses have shown that consumption of vegetables from the Brassicaceae family are inversely associated with the risk of many cancers, including cancers of the breast^3^, colon^4^, gastro-intestinal tract^5^, lung^6^, pancreas^7^ and prostate^8^. Although Brassica vegetables contain high levels of several nutrients and phytochemicals including vitamins C, E and fibre, it has been suggested that the main preventive role of Brassicaceae may not be attributed to those molecules^9^. Instead, studies have shown that glucosinolates (which upon hydrolysis produce isothiocyanates such as sulforaphane and 3,3′-diindolylmethane (DIM)), are unique to crucifers and are thought to explain the cancer preventive role of Brassicaceae^10^,^11^,^12^. Transcriptomic and proteomic studies demonstrate that the intake of Brassica vegetables affects many different pathways (reviewed in ref. 13). It is unlikely that this effect is achieved by only one component, but rather, may be dependent upon interaction of several bioactive molecules.

MicroRNAs are small RNA molecules that have the ability to control the expression of numerous messenger RNAs^14^, and their aberrant expression has been linked to multiple diseases^15^ (http://210.73.221.6/hmdd). Liang *et al*. recently demonstrated in mice that *Brassica oleracea* microRNAs survive the passage through gastrointestinal tract following digestion, and can be detected in the blood as well as other organs (e.g., stomach, intestine and spleen)^16^. Nevertheless, the role of food-related microRNAs and their ability to impact cross-species mRNA regulation remain highly debated, and there is a need for well-designed studies^17^.

In the current study, we established the detectability of Brassica microRNAs in human blood both in a large cohort and in a dose-controlled randomized trial. In addition, we performed *in vitro* experiments showing that Brassica microRNAs can regulate the expression of key human cancer-related genes.

## Results

### *Brassica oleracea* microRNAs detection in blood

A complete list of 64 microRNAs assigned to *Brassica oleracea* is available at mirNEST (http://rhesus.amu.edu.pl/mirnest/copy/home.php) and listed in Supplementary Table 1.

We decided to focus our analysis on lung cancer, the main cause of cancer-related death worldwide^18^, for which a preventive role for Brassicaceae consumption has been described^6^. To prioritize broccoli microRNAs for validation studies, we predicted their targets, and we cross-referenced them with the genes significantly and frequently upregulated in lung cancer, resulting in 193 upregulated targets (Supplementary Table 2). Summary data for 8 microRNAs prioritized according to number of upregulated targets and predicted binding energy is presented in Supplementary Table 3. With the exception of miR160 and miR168, the selected microRNAs are specific for *Brassica oleracea*. In human diet, flowers are the most frequently consumed broccoli part, followed by stem and, less frequently, leaves. Given the difference in consumption behaviour, we quantified the expression of 8 selected microRNAs in leaf, stem and flower samples. To account for differences in microRNA expression influenced by plant stage of development and environmental stimuli, we selected two “organic” and two conventional sources of broccoli obtained from four different vendors. We tested both the precursor and mature forms of the microRNAs. Figure 1 highlights the variability of microRNA expression among different parts of the same broccoli plant. Surprisingly, there is high expression variability in the same part of the broccoli plant purchased from different vendors (Supplementary Fig. 1). It is intriguing that samples from Vendor 1 show little or no expression of precursor microRNAs while Vendor 3 samples have a high expression of precursor (Supplementary Fig. 2). Since mature microRNAs have less variability than precursor ones, we focused the remaining analyses on the mature form of microRNAs. The mature microRNAs with the highest expression across samples and in particular in the flower part included: miR160, miR2673 and miR917. Finally, we selected miR160 and miR2673 for further analyses since they are predicted to target the highest number of genes upregulated in lung cancer (Supplementary Table 3).

### Brassica microRNAs are detectable in human serum from a retrospective nutrigenomics study

Next, we tested the detectability of miR160 and miR2673 circulating in blood of human subjects with regular consumption of broccoli, and evaluated the variability in the amount of detected microRNA. We compared the serum levels of 52 healthy individuals from an existing cross-sectional study (Supplementary Fig. 3), 26 of which were labelled as consumers (i.e., reported consumption of at least one portion of cruciferous vegetables per day) and 26 non-consumers, which included individuals who did not regularly consume cruciferous vegetables. Individuals were matched for age and ethnicity, and the sex ratio in each group was 1:1 (Supplementary Table 4). There is a significant difference in amount of detected microRNAs in blood of individuals with regular daily consumption of cruciferous vegetables versus non-consumers (p < 0.005 for both microRNAs; Fig. 2a), confirming our ability of detecting Brassica microRNAs. Moreover, miR2673 showed a tighter grouping compared to miR160, likely due to the former being specific only for *Brassica oleracea* vegetables. One individual in the consumption group did not have either microRNA detectable. This individual did not report any underlying health or disease concerns, and as the samples were anonymized, it was not possible to identify whether this may have been incorrect reporting of the usual diet or another factor, such as a metabolic anomaly. It is also intriguing that there was variability in the non-consumption group, possibly due to incomplete reporting of the diet (the food frequency questionnaire used to capture diet consisted of ‘yes/no’ answers as well as frequency of consumption and the questions include ‘most’ but not ‘all’ Brassica species; see Methods). Besides the food source effect discussed above, food preparation may have also influenced microRNA content. To address this variability, we first investigated how cooking affects broccoli microRNA expression, and then performed a controlled, dietary intervention to analyse dose-dependent effect in a randomized clinical trial (Supplementary Figure 4).

### Cooking procedures affect broccoli microRNAs expression

To confirm that raw broccoli is an optimal source of microRNAs, we investigated the effect of 7 common cooking methods on miR160 expression. As shown in Fig. 2b, baking and microwaving, as well as the procedure of pouring hot water on raw broccoli and letting it rest for 3 minutes result in the highest amount of microRNA. Increasing the time the broccoli remained in hot water reduced the amount of detectable microRNA. The most significant reduction in microRNA was observed when broccoli was blended or steamed (p < 0.0001). Thus, raw or shortly cooked broccoli provides the best source of microRNAs, and potentially strongest health benefits. Interestingly, long exposure to hot water, steaming and blending degrade microRNAs’ integrity, reducing the potential benefits.

### Brassica microRNAs are detectable in human serum in a serving-controlled randomized trial

We then ran a controlled intervention study, with a pre-defined daily broccoli serving and tracked dietary intake. The goal was to identify a dose-dependent relationship between broccoli consumption and circulating broccoli microRNAs. For this purpose, we recruited 19 healthy volunteers that followed one of three dietary interventions described in the Methods section and Supplementary Fig. 4. At the beginning of the study, all individuals refrained from eating Brassicaceae for one week, subsequently ate 80 g of raw broccoli daily for one week and in the last week the three experimental groups were: six individuals eating 160 g of broccoli per day, seven eating 80 g per day, and six abstaining from eating Brassicaceae. We observed that the amount of circulating miR160 and miR2673 was significantly decreased after one week of fasting from Brassicaceae (p < 0.01, Fig. 2c), while it significantly increased again after the ingestion of 80 g of broccoli per day (p < 0.01). Doubling the daily dose of broccoli further significantly increased the presence of the microRNA (p < 0.0001), while refraining from eating Brassicaceae was associated with a significant decrease (p < 0.01). Sequencing of the PCR products confirmed amplification of the microRNA and its specificity (as shown in Supplementary Table 5). hsa-miR21 was included as a negative control and, as shown in Fig. 2c, there was no change in its detection during the entire experiment. Individuals who continued eating 80 g of broccoli/day maintained a similar amount (p = 0.37 for miR160 and p = 0.10 for miR2673) but showed a small decrease in the detectable circulating microRNAs, suggesting a possible tendency to plateau after a longer exposure to a constant amount of broccoli. We thus conclude that broccoli microRNAs can be detected in serum in dose and time dependent manner.

### Brassica microRNAs target human genes *in vitro*

Since several epidemiologic studies have demonstrated preventive role of Brassica vegetables consumption on multiple cancer types, we set out to investigate whether miR160 downregulates genes that are significantly and frequently upregulated in non-small-cells lung cancer (NSCLC). We have focused on lung cancer as it remains the main cause of cancer-related death worldwide^18^, and specifically on NSCLC since it accounts for about 80–85% of all lung cancer cases^19^.

We have selected two NSCLC cell lines with the highest expression of at least one of the genes identified as putative broccoli miRNA targets. We then transfected the two cancer cell lines with miR160 mimic, and measured the potential downregulation of the targets. Figure 3 shows that 8 out of 9 tested genes were significantly downregulated by miR160 transfection ((p < 0.05); MCM5 was not changed). Supplementary Figure 5 shows the amount of transfected miR160 per cell line, while Supplementary Table 6 lists p-values for comparisons of all samples against AllStars Negative Control. There was no significant difference between AllStars Negative Control, transfection reagent and not treated cells (Supplementary Table 6). NCBP2 and SHMT2 were significantly reduced both as transcript and protein, while MTHFD2 was reduced as transcript but not protein, after miR160 transfection (Supplementary Figure 6). Human microRNA regulation of CDC6 has already been described as a mechanism of prevention of lung cancer formation^20^, while PYCR1 and MTHFD2 have been shown to be required for breast tumorigenesis *in vitro*^21^.

### miR160 complements bioactive compounds

As several compounds found in Brassica vegetables had been implicated having anticarcinogenic effects on tumor cells, we decided to test whether molecular targets can be uniquely affected by miRNAs or whether it is a combined effect of Brassica microRNAs and natural compounds. However, the only publicly available dataset suitable to test this hypothesis is a study where gastric biopsies were collected before and after ingestion of high glucosinolate (HG, enriched in sulforaphane) or regular broccoli^22^. As reported, ten probes were downregulated and 20 were upregulated after ingestion of HG broccoli while 21 were downregulated and two were upregulated after ingestion of regular broccoli; the overlap of the two sets comprised 8 probes (201170_s_at, 209674_at, 209750_at, 209803_s_at, 225768_at, 225840_at, 228846_at, 244677_at).

We decided to test 11 genes, 4 deregulated after HG broccoli exposure, 3 deregulated after regular broccoli exposure and 4 in common between the two sets, in a gastric cell line expressing all these targets, MNK45. We transfected the cells with miR160 mimic, and treated them with sulforaphane or DIM, and for each treatment, we tested the change in expression of the selected genes. DIM was included in the experiment because it is one of the two isothiocyanates present in Brassicaceae, together with sulforaphane, most frequently studied for their anticancer properties^10^. As shown in Fig. 4, the two genes upregulated in HG gastric biopsies are also upregulated after treatment with sulforaphane while only one (AKR1C2) is upregulated after treatment with DIM. Of the remaining 9 downregulated genes, 6 were deregulated solely by miR160, one by miR160 and sulforaphane (DUSP4) and one by miR160 and DIM (FOS). Student’s t test p-values calculated for each gene in DIM, sulforaphane or miR160 treatment against not treated cell lines are listed in Supplementary Table 7.

These results indicate that half of the tested genes would not validate if only chemical compounds are considered for biological activity of Brassica vegetables. This highlights the complementary effects of microRNAs and active compounds present in broccoli, and emphasizes the importance of considering multiple components and mechanisms when studying the effect of diet on health.

## Discussion

After Zhang *et al*. first publication reporting plant microRNAs detected in human blood^23^, several researchers tried to replicate and further address those findings. While the results remain debated, it is clear that these studies need to be properly planned and well controlled to provide meaningful results.

Three studies failed to detect plant microRNAs in plant-fed organisms: Witwer *et al*. detected a variable amount of plant microRNAs in blood of only two *Macaca nemestrina* with one PCR technique and a low amount with two others^24^; Snow *et al*. failed to detect plant microRNAs in blood of athletes that reported eating fruit for breakfast at the day of blood collection, and detected low amounts in mice plasma and tissues (when mice were fed fresh avocado instead of processed food)^25^; Dickinson *et al*. detected very low reads in mice plasma and liver with deep sequencing^26^, but the technique used has been questioned^27^. Two other publications suggested that the detection of plant microRNAs in human datasets can be due to contamination from other samples rather than from the real presence of such microRNAs^28^,^29^. Nevertheless, more groups are confirming the findings from Zhen *et al*. after performing more accurate and directed studies. Wang *et al*. set up a more accurate method to detect exogenous microRNAs in deep sequencing data and succeeded in identifying a higher amount of such molecular species than other studies^30^. Liang *et al*. demonstrated the presence of plant microRNAs in different mice tissues and provided a very useful time curve of appearance and disappearance of the microRNAs^16^. Similarly, Yang *et al*. demonstrated that plant microRNAs are detectable in mice serum and urine at levels proportional to the amount of microRNA present in the plant fed to the animal, while a significant amount of the synthetic form of the microRNA fed to the animals would barely increase the detection of the molecule and would be cleared fast when injected in the tail vein^31^. The same group also demonstrated that the amount of plant microRNAs increases when there is a pathological or induced alteration in intestinal permeability^32^. Interestingly, studies on exogenous microRNAs are not limited to microRNAs detection: Zhou *et al*. demonstrated the ability of the plant microRNAs to reach blood and lung in mice, and to suppress Influenza A viruses replication^33^; Mlotshwa *et al*. modified mice tumor suppressor microRNAs to molecularly resemble plant microRNAs, and after feeding them to mice detected a significant reduction in tumor burden^34^; Chin *et al*. demonstrated a correlation between amount of plant microRNAs in human blood and protection from breast cancer, detected a proportional amount of plant microRNAs in breast tumor tissue and proved the ability of miR-159 to reduce cell growth *in vitro* and tumor weight *in vivo*^35^.

In this context, our findings provide evidence that microRNAs should be included in functional studies alongside bioactive compounds in order to establish a more comprehensive understanding of the underlying mechanisms of the protective effects of vegetables and fruit on human health. Demonstrating the molecular ability of plant-derived microRNAs to control human genes *in vitro*, suggests that we cannot ignore these short molecules when considering epidemiological effects of edible plants.

Importantly, our data obtained from large population study and a dose-controlled randomized trial proved strong dose-dependent correlation of broccoli microRNAs detected in human serum. Our randomized trial also further highlights the need for properly controlled studies to investigate molecular effects of dietary intakes, in order to reduce the impact of confounding factors always present when dealing with individual lifestyle habits, source and preparation variations. Our results suggest that the amount of circulating Brassica microRNAs significantly increases with the increment of Brassica plant intake. It also indicates that the expression saturates if maintaining the same number of servings, suggesting a possible mechanism of the human body adaptation to a constant amount of plant-derived microRNA exposure that needs further investigations with longer exposure times.

Finally, well-designed intervention studies evaluating other food and microRNAs are necessary to continue to thoroughly address the detectability and possible roles of exogenous microRNAs circulating in human blood on the regulation of gene expression and their connection to human health.

## Methods

### microRNAs targeting and prioritization

*Brassica oleracea* microRNAs were obtained from miRNEST 2.0 (http://rhesus.amu.edu.pl/mirnest/copy/; downloaded Sep. 15^th^, 2014). To establish if the existence of any of these microRNAs is already experimentally validated, we searched for *Brassica oleracea* microRNAs in PMRD version 1^36^ (http://bioinformatics.cau.edu.cn/PMRD/). Since only bol-miR824 has been experimentally validated, we have included it in the subsequent analysis independently of further prioritization.

Each mature microRNA sequence was cross-referenced against the entire miRNEST set to identify species specificity.

Targeting of Brassica microRNAs to human genes was predicted using the Probability of Interaction by Target Accessibility (PITA) algorithm version 6^37^ against human 3′ UTR (UCSC hg19, GRCh37, http://hgdownload.cse.ucsc.edu/downloads.html#human). As described by the authors, putative hits were defined by the recommended ΔΔG threshold of −10 kcal/mol·K. These searchable hits are available to the public through the mirDIP 2 portal (http://ophid.utoronto.ca/mirDIP).

To prioritize microRNAs to test in our subsequent analyses, we surveyed CDIP version 1 (http://ophid.utoronto.ca/cdip) for genes deregulated in lung cancer and retained those that were upregulated in more than 10 studies. We then selected for our analysis *Brassica oleracea* microRNAs targeting the highest number of these genes and with a more stringent thermodynamic energy threshold than the one suggested by PITA authors (lower than −15 kcal/mol·K).

### Plant samples and extraction

As a representative *Brassica oleracea* edible plant, we chose broccoli, a plant found in worldwide diets. Broccoli plants were obtained from four different vendors in Toronto: Loblaws (1, http://www.loblaws.ca), Metro (2, http://www.metro.ca), Costco (3, http://www.costco.ca) and Sobeys (4, https://www.sobeys.com). Plants from Loblaws and Metro were “organic” while the latter two samples were from conventional sources. A small cube or square (3 mm per dimension) was sampled from flowers (at the very top of the plant), stems (1 cm below the flower crown) and the centre of leaves.

Samples were further cut with small scissors and then resuspended in 1 ml of Tri-reagent (BioShop, Canada). After letting the solution stand for 10 minutes in ice, samples were spun at 13,000 g for one minute using DNA IQ Spin Baskets (Promega, Madison, WI, USA) to separate plant matter. 500 μl of flow through solution was collected and used for RNA extraction following the first part of manufacturer’s protocol. When aqueous phase was collected, the extraction proceeded using RNeasy Mini Kit (Qiagen, Limburg, Netherlands) according to manufacturer’s protocol.

To test the effect of cooking procedures on microRNAs, we performed 3 rounds of different cooking procedures using one head of broccoli from Costco for each of them. The procedures were: baked, wrapped in aluminum foil, for 10 minutes at 175 °C; steamed 8 minutes; microwaved for 5 minutes in water at 750 W; pan fried 5 minutes in water; boiled 5 minutes; poured hot water in a container above raw broccoli and let sit for 3, 5 and 10 minutes; blended in water for 3 minutes using Magic Bullet. Samples were put in 500 μl of RNAlater (Life technologies) and extracted as described above. 1 ml of water was also collected from steamed, boiled and poured samples, spun at 3,000 g for 10 min, 500 ul of supernatant were removed and 1 ml of Tri-reagent was added to proceed according to the above protocol.

Broccoli plants for the randomized trial were purchased at Costco, twice per week. We used packages of broccoli heads (same vendor and batch) to ensure the consumption of the same part of the plant by all study participants in all time points.

### Human samples and extraction

To test the presence of Brassica microRNAs in serum of young individuals eating broccoli, we selected 40 individuals from the Toronto Nutrigenomics and Health (TNH) Study (n = 1,631). The TNH Study is a cross-sectional examination of young men and women aged 20–29 years who were recruited from the University of Toronto campus between October 2004 and December 2010^38^. The study was approved by the University of Toronto Ethics Review Board and all experiments were performed in accordance with relevant guidelines and regulations. Subjects completed a 1 month 196-item semi-quantitative Toronto-modified food frequency questionnaire (FFQ), a general health and lifestyle questionnaire, a physical activity questionnaire, and provided a fasting blood sample. Pregnant or breastfeeding women as well as individuals who were fasting for religious reasons were excluded from the study. Subjects were divided into high-cruciferae consumers (at least one serving per day) and low-cruciferae consumers (0 servings per day) according to their broccoli intake as reported in the FFQ. We collected a serum aliquot of 200 μl for each of them and the summary features for each group is listed in Supplementary Table 4.

Moreover, we performed a controlled prospective study: volunteers were included upon providing written informed consent (study approved by University Health Network Research Ethics Board, REB 13-7077 AE. All experiments were performed in accordance with relevant guidelines and regulations. We included only volunteers that were not allergic to broccoli). 15 ml of blood were collected in ACD before any intervention (time zero); after one week of abstaining from eating Brassicaceae (where individuals refrained from eating *Brassica oleracea* vegetables, time 1); after one week of consumption of 80 g of broccoli per day (time 2) and at the end of the subsequent week where individuals were split in 3 groups (time 3, one group was consuming 160 g of broccoli per day, one group was consuming 80 g of broccoli per day and one group was not eating broccoli). Supplementary Figure 2 depicts the collection’s protocol. During the two weeks where individuals were eating broccoli, they were asked to avoid any other vegetables from the Brassica family. Individuals were given pre-packaged daily doses of broccoli twice per week (3 doses on Monday and 4 doses on Thursday).

Blood was centrifuged at 2,000 g for 10′ and 3 serum aliquots of 200 μl each were collected and stored at −80 °C. RNA extraction was performed in one of the 3 aliquots using Tri-reagent (BioShop, Canada) and RNeasy Mini Kit (Qiagen, Limburg, Netherlands) according to manufacturer’s protocol as described above.

### Real Time PCR

RNA for each sample was reverse transcribed using miScript II RT Kit (Qiagen) following manufacturer’s instructions. Resulting cDNA was diluted 1:10 and used to perform Real Time PCR using miScript SYBR Green PCR Kit (Qiagen) following manufacturer’s protocol. To test mature microRNAs expression we used the (reverse) Universal Primer included in the kit and designed our own forward, while for precursor microRNAs and genes expression we designed both primers (all listed in Supplementary Table 8). Moreover, to confirm the effect of miR160 or Brassica compounds on genes reported as deregulated in Gasper *et al*.^22^, we designed primer pairs for 11 such genes. We used Primer Design tool in the Visual OMP software package (version 7.6.58 DNA Software Inc., Ann Arbor, MI, USA) under conditions at 55 °C, 0.05 M NaCl, 0.002 M MgCl_2_, at 1 × 10^−7 ^M concentration and primers were selected based on percent bound. Custom primers were simulated *in silico* with Simulation tool included in Visual OMP package (DNA Software Inc.) to ensure a high specificity to low noise ratio. All Real Time PCRs were run in a LightCycler 480 System (Roche). In all Real Time PCRs, we calculated expression using geometric mean of reference genes. In cell lines, values were normalized on non-treated (MNK45 cell lines) or AllStars transfected cells (H2170 and H2290). In MNK45 case, expression was log2 transformed to make the values comparable to the ones collected in the literature.

To ensure specificity of the broccoli microRNA PCR products in human blood, we cloned the amplified PCR products of miR-160 and miR-2673 into the pUCM-T cloning Vector (Bio Basic Inc) using DH5α-competent cells. The plasmid was purified using EZ-10 Spin Column Plasmid DNA mini-preps kit as per the manufacturer’s direction. Sequences were confirmed by Sanger sequencing (The Centre for Applied Genomics, Sick Kids Hospital, Toronto) and computationally aligned using blastn (http://blast.ncbi.nlm.nih.gov/Blast.cgi?PROGRAM=blastn&PAGE_TYPE=BlastSearch&LINK_LOC=blasthome).

### Cell lines and transfection

Non-small cell lung cancer and gastric cell lines with the highest expression of the genes of interest were selected based on data collected from CCLE (http://www.broadinstitute.org/ccle/home downloaded on September 29, 2012).

H2170 and H2290 lung cancer cell lines were kindly provided by Dr. Ming Tsao (University Health Network) while MNK45 gastric cancer cell lines were kindly provided by Dr. Morag Park (McGill University). All cell lines were cultured in RPMI 1640 (Invitrogen, Life technologies, Grand Island, NY, USA) supplemented with 10% fetal bovine serum (Invitrogen) and 1% streptomycin/penicillin (Sigma-Aldrich, St. Louis, MO, USA) at 37 °C and 5% CO_2_.

All cell lines were transfected with 50 nM miR160 mimic or 50 nM AllStars Negative Control (Qiagen) and siPORT NeoFX Transfection Agent (Life technologies) according to manufacturer’s protocol. Each well was harvested after 48 hours and RNA was extracted as described above.

Gastric cell lines were also treated with Sulforaphane, (Sigma-Aldrich, at IC50 20 uM), diindolylmethane (Sigma-Aldrich, DIM) (at IC50 100 uM) and DMSO (1%).

### Western Blotting

Cells were homogenized in a RIPA buffer supplemented with protease and phosphatase inhibitor cocktails (Roche). The homogenates were centrifuged at 13,000 r.p.m for 10 minutes, and the supernatants were used as whole-cell lysates. Protein concentration was assessed by Bio-Rad BCA protein assay. 30 ug of protein lysate was separated by SDS-PAGE and then transferred on to a PVDF membrane. The membranes were probed with primary anti-CDC6 (Bethyl Laboratories Inc., cat. A302-487A-T-1), anti-NCBP2 (Bethyl Laboratories Inc., cat. A302-553A-T), anti-SHMT2 (Cell Signaling, cat. 12762), anti-MTHFD2 (Cell Signaling, cat. 41377) – all at 1:1,000 dilution – or anti-actin (Santa Cruz Biotechnologies) – at 1:500 dilution – for 1 h. Membranes were washed and then incubated with HRP-conjugated donkey anti-rabbit (Santa Cruz Biotechnologies) at 1:5,000 dilution or HRP-conjugated donkey anti-goat (Santa Cruz Biotechnologies) at 1:10,000 dilution. Protein was detected with Western Lightning Plus-ECL (Perkin Elmer), and analyzed using ImageJ Software ver. 1.50 (NIH, USA).

### Gene expression dataset and statistical analysis

A publicly available dataset that measured gene expression data before and after ingestion of Brassicaceae was used for our analysis, which describes gene expression changes in gastric mucosa before and after ingestion of regular or high glucosinolate (enriched in sulforaphane) broccoli (in the paper we refer to these samples as to “regular” and “HG”)^22^. We have created a list of deregulated genes using supplementary data from this study.

Statistical analyses were performed using GraphPad PRISM 6.05. MicroRNA transfected samples were compared to samples treated with AllStars Negative Control using t-test. In gastric cell lines, microRNA transfected or compound treated cells were compared to not treated using t-test. Samples from different cooking procedures were compared to raw broccoli using one-way ANOVA and multiple comparisons. Samples from individuals eating high amount of Brassicaceae per day were compared to samples eating low amount with Mann-Whitney test. Samples from different time points of the controlled broccoli study were compared among each other using two-way ANOVA and multiple comparisons.

## Additional Information

**How to cite this article**: Pastrello, C. *et al*. Circulating plant miRNAs can regulate human gene expression *in vitro*. *Sci. Rep*. **6**, 32773; doi: 10.1038/srep32773 (2016).

## Supplementary Material

Supplementary Information

## Figures and Tables

**Figure 1:** Expression of 8 microRNAs in three plant parts from 4 vendors. The first three rows show expression of mature microRNAs for stems, leaves and flowers in this order, while rows 4 to 6 show expression of precursor form of microRNAs for stems, leaves, and flowers in this order. Each column represents a different broccoli microRNA (all listed in the upper part of the figure). Each panel shows expression of a specific broccoli microRNA for a specific plant part from four different vendors (45° hash pattern bar vendor 1, 135° hash pattern bar vendor 2, white bar vendor 3 and gray bar vendor 4).

**Figure 2:** Detection of miR160 and miR2673. (**a**) Amount of microRNA detected in sera collected in an epidemiological study, comparing persons eating a high amount (at least one serving, i.e., 80 g) or a low amount (0 servings) of Brassicaceae per day. p-values from ANOVA are shown. (**b**) Expression of miR160 in cooked broccoli samples. Broccoli was cooked using 7 different techniques, and in one case (poured) using three different time points (3 minutes P_3, 5 minutes P_5 and 10 minutes P_10). Expression was normalized to raw broccoli. p-values (ANOVA): **0.01–0.001, ***0.001–0.0001, ****<0.0001. (**c**) Expression in plasma of individuals eating no Brassicaceae (T1 and T3 0 g), 80 g of broccoli per day (T2 and T3 80 g), 160 g of broccoli per day (T3 160 g). p-values were calculated using the Mann Whitney test.

**Figure 3:** Effect of miR160 transfection on targets expression. Ratio of expression of tested genes after transfection of miR160 in two NSCLC cell lines compared to expression in negative control (AllStars, scrambled sequence). siPORT = transfection reagent. NT = not treated. p-values (t-test): *0.05–0.01, **0.01–0.001.

**Figure 4:** Heatmap of deregulated genes in gastric biopsies or gastric cancer cell line. The figure shows fold change for 11 genes and miR160 in 5 set of samples. High glucosinolate (HG) and regular represent samples from gastric biopsies after ingestion of HG (enriched in sulforaphane) or regular broccoli as per Gasper *et al*.^22^, and fold change data is collected from the same paper. Sulforaphane, DIM and miR160 refer to MNK45 cell line treated with each of the named molecules, and fold change was measured by real time PCR (log transformed to be comparable to Gasper *et al*. fold change). Blue blocks represent downregulated genes, red to green blocks upregulated ones. Grey blocks are missing values from Gasper *et al*. paper.
